The article "The Effect of Different Degrees of Ankle Dorsiflexion Restriction on the Biomechanics of the Lower Extremity in Stop-Jumping" was published in 2024. Journal: Appl Bionics Biomech.

# The Effect of Different Degrees of Ankle Dorsiflexion Restriction on the Biomechanics of the Lower Extremity in Stop-Jumping

**DOI:** 10.1155/2024/9079982

**Published:** 2024-08-28

**Authors:** Zanni Zhang, Datao Xu, Xiangli Gao, Minjun Liang, Julien S. Baker, Yaodong Gu

**Affiliations:** ^1^ Faculty of Sport Science Ningbo University, Ningbo, China; ^2^ Faculty of Engineering University of Pannonia, Veszprem, Hungary; ^3^ Department of Radiology Ningbo No. 2 Hospital, Ningbo, China

## Abstract

**Purpose:**

The functional status of the ankle joint is critical during dynamic movements in high-intensity sports like basketball and volleyball, particularly when performing actions such as stopping jumps. Limited ankle dorsiflexion is associated with increased injury risk and biomechanical changes during stop-jump tasks. Therefore, this study aims to investigate how restricting ankle dorsiflexion affects lower extremity biomechanics during the stop-jump phase, with a focus on the adaptive changes that occur in response to this restriction. Initially, 18 participants during stop-jumping with no wedge plate (NW), 10° wedge plate (10 W), and 20° wedge plate (20 W) using dominant leg data were collected to explore the relationship between limiting ankle mobility and lower extremity biomechanics. Following this, a musculoskeletal model was developed to simulate and calculate biomechanical data. Finally, one-dimensional parametric statistical mapping (SPM1D) was utilized to evaluate between-group variation in outcome variables using a one-way repeated measures analysis of variance (ANOVA).

**Results:**

As the ankle restriction angle increased, knee external rotation angles, knee extension angular velocities, hip extension angle, and angular velocity increased and were significantly different at different ankle restriction angles (*p*  < 0.001 and *p*=0.001), coactivation of the peripatellar muscles (BF/RF and BF/VM) increased progressively, and patellofemoral joint contact force (PTF) increased progressively during the 3%–8% phase (*p*=0.015). These results highlight the influence of ankle joint restriction on lower limb kinematics and patellofemoral joint loading during the stop-jump maneuver.

**Conclusion:**

As the angle of ankle restriction increased, there was an increase in coactivation of the peripatellar muscles and an increase in PTF, possibly because a person is unable to adequately adjust their body for balance when the ankle valgus angle is restricted. The increased coactivation of the peripatellar muscles and increased patellofemoral contact force may be a compensatory response to the body's adaptation to balance adjustments.

## 1. Introduction

Termination tasks are common movements in high-intensity sports such as basketball and volleyball. These maneuvers involve sustained starts, stop-jumping, and rapid lateral movements [1, 2, 3]. Among these, the stop-jumping technique is fundamental in showcasing an athlete's body control and explosiveness during gameplay in sports such as basketball and volleyball. Previous authors have thoroughly described stop-jumping, comprising the jump, rapid stop (horizontal landing phase), and subsequent jump [4, 5]. The ankle joint plays a pivotal role in executing the stop-jumping maneuver, serving as the primary joint for power transmission to the ground. Studies have emphasized the critical relationship between ankle joint function and sports injuries [6]. Limited ankle mobility heightens injury risks during stop-jumping [7, 8]. Analyzing lower extremity biomechanics can aid in predicting and preventing sports-related injuries [9]. Thus, comprehending the impact of ankle mobility on stop-jumping and its correlation with lower limb biomechanics is imperative for athletes' well-being and performance.

The article "The Effect of Different Degrees of Ankle Dorsiflexion Restriction on the Biomechanics of the Lower Extremity in Stop-Jumping" was published in 2024. Journal: Appl Bionics Biomech.

In a study analyzing the kinematics and kinetics of ankle injuries in basketball players, researchers observed increased stress on the lower extremity during stop-jumping [10]. This underscores the importance of understanding the biomechanics involved in such maneuvers, with foot and ankle mobility being critical factors [11]. Optimal foot and ankle function is essential for effective force transfer, stability, and injury prevention during these dynamic activities [12]. Previous research has established that increasing the ankle's initial contact angle and its range of motion (ROM) in a single leg enhances energy dissipation in the lower limb joints and decreases peak forces on the anterior cruciate ligament (ACL). This reduction in peak forces subsequently lowers impact loads on the lower limb joints, thereby diminishing the risk of injuries, including ACL injuries [13, 14]. In contrast, restricted mobility in the foot and ankle can substantially impair biomechanical performance and elevate the risk of injuries [15, 16, 17]. Research has shown that reduced ankle mobility can lead to biomechanical alterations affecting jumping ability [16]; reduced dorsiflexion angles have been observed in individuals classified as copers (during drop-landing tasks and prelanding tasks) and those with chronic ankle instability (during drop landing and forward jump followed by a landing task) when compared to healthy participants [18]; healthy female athletes, for example, typically exhibit greater dynamic functional range of motion (DFROM) during jump landings. Decreased ankle DFROM is associated with a heightened risk of injury during jump-landing tasks [17]. It is worth noting that in patients with mild flatfoot, the addition of arch support to the heel pad does not significantly affect ankle and metatarsophalangeal joint angles during unplanned gait termination [19]. Previous studies have confirmed that wearing athletic shoes designed to create an unstable condition significantly affects the ROM of ankle dorsiflexion. The increased dorsiflexion facilitated by this unstable footwear may enhance balance and proprioception. However, the augmentation in ROM must be carefully managed to prevent excessive strain or overuse injuries to the ankle and its associated structures [20].

The article "The Effect of Different Degrees of Ankle Dorsiflexion Restriction on the Biomechanics of the Lower Extremity in Stop-Jumping" was published in 2024. Journal: Appl Bionics Biomech.

Research indicates that modifying the ankle's initial contact angle can significantly reduce the risk of knee injuries [21], while decreasing ankle valgus can lower the likelihood of developing patellar tendinopathy [22]. Previous studies have found a correlation between reduced ankle dorsiflexion and the occurrence of tendinopathy during drop and spike landings. Additionally, jumping athletes demonstrated diminished knee joint power and work during volleyball approach and drop landings [23]. These modifications can prompt adaptive responses in the peripatellar muscles, enhancing their capacity to handle increased loads. For instance, the peripatellar muscles may hypertrophy or become more adept at absorbing impact to compensate for reduced ankle mobility. Therefore, studying how ankle mobility impacts knee adaptations can provide valuable insights into the biomechanical alterations that athletes undergo when faced with limitations in ankle mobility.

Previous studies have highlighted the significance of foot and ankle mobility in enhancing exercise performance and mitigating injury risks [24, 25, 26, 27]. Nevertheless, modeling the impact of restricted ankle mobility on lower extremity biomechanics remains an underexplored area. Comprehending how limited ankle mobility influences lower extremity biomechanics can provide valuable insights into compensatory mechanisms, alterations in exercise strategies, and potential injury risks associated with such limitations. Our study hypothesized that increased limitations in ankle dorsiflexion mobility would induce adaptive changes in the body to compensate for these restrictions.

## 2. Methods

### 2.1. Participants

In this study, a priori power analysis was performed utilizing G-power software (version: 3.1.9.7; Henry University of Düsseldorf, Düsseldorf, Germany) to assess the sample size required for experimental design [28]. Using one-way repeated measures analysis of variance (ANOVA) with statistical power and significance levels fixed at 0.80 and 0.05 [29], the number of repeated measures was calculated to be seven and the number of groups comprising three. The results showed that to achieve a medium effect size of 0.5, a sample size of at least 18 participants was required.

The article "The Effect of Different Degrees of Ankle Dorsiflexion Restriction on the Biomechanics of the Lower Extremity in Stop-Jumping" was published in 2024. Journal: Appl Bionics Biomech.

This study recruited 18 male amateur basketball and volleyball players from Ningbo University; prior to data collection, all participants were thoroughly informed about the study's purpose, procedures, conditions, and requirements. Detailed study information was provided in a consent form, which was signed by each participant. The study received approval from the Ethics Committee of Ningbo University (Protocol Code: RAGH20231009).

### 2.2. Data Collection Procedures

All tests were conducted in the Sports Biomechanics Laboratory at the Research Academy of Grand Health, University of Ningbo. The Vicon motion capture system (Oxford Metrics Ltd., Oxford, UK), featuring eight cameras, was employed to capture the kinematic data of participants during the stop-jumping task. The sampling frequency was set at 200 Hz [30, 31]. During the stop-jumping task, the force platform (AMTI, Watertown, Massachusetts, USA) was set to a sampling frequency of 1,000 Hz to collect kinetic data. Both experimental setups were synchronized. The initial contact was defined as the point at which the vertical ground reaction force exceeded 10 N [32]. All participants wore tight-fitting shorts and shirts. Consistent with previous research, 38 spherical reflective markers with a diameter of 12.5 mm were affixed to each participant to identify movement patterns during each trial [33]. Surface EMG for non-invasive assessment of muscles (SENIAM) guidelines were followed when placing the electromyography (EMG) sensors [34]. Eight EMG sensors (Delsys, Boston, MA, USA) were attached to the muscle bellies of the soleus (SOL), medial gastrocnemius (MG) and lateral gastrocnemius, tibialis anterior (TA), rectus femoris (RF), vastus lateralis, vastus medialis (VM), and biceps femoris (BF) to measure muscle activation. Reflective markers were placed at specific anatomical landmarks on the body, as shown in Figure 1(a), and EMG was placed at specific anatomical markers on the body, as shown in Figure 1(b).

Participants began by warming up on a treadmill for 10 min at a speed of 8 km/hr. Following this, they performed stretching exercises to ensure they could perform at their maximum potential during the experiment. Participants wore tight-fitting shirts and shoes in accordance with the formal experimental requirements. Each participant was given three opportunities to familiarize themselves with the testing movements. After the warm-up phase, participants were thoroughly acquainted with the experimental conditions and procedures before starting the full testing protocol. Participants were instructed to stand on the force plate to collect static coordinates before formal data collection began. During this time, each participant's feet were aligned parallel to the *y*-axis, with their gaze fixed forward until the static data collection period concluded [31].

The article "The Effect of Different Degrees of Ankle Dorsiflexion Restriction on the Biomechanics of the Lower Extremity in Stop-Jumping" was published in 2024. Journal: Appl Bionics Biomech.

To collect biomechanical data, each participant initially positioned their left foot forward and their right foot back. Upon hearing a command, they immediately stepped forward with their right foot, with the left foot following the right foot as the right foot landed, and then performed a stop-jumping task. Three different takeoff angles were utilized in our study, which were performed on flat ground with no wedge (NW), 10° wedge (10 W), and 20° wedge (20 W) board, respectively.  Figure 1(c) illustrates the plyometric jumping movement. Participants were instructed to jump as high as possible vertically [35, 36, 37]. The data collected exclusively focused on the participants' right legs, with all individuals having their dominant limb as the right leg. The dominant limb was identified as the preferred leg for kicking a ball [33].

During the stop-jumping task, if participants were observed to exhibit any nonvertical jumps or sliding motions, the trial was recorded as a failure. Seven successful datasets were collected using the dominant leg, equivalent to 21 datasets per participant across the three different takeoff angles. There was a 1-min rest period between each test and a 5-min rest period between jumps at each takeoff angle to prevent participants from becoming overly fatigued. This was crucial as individual fatigue could lead to inaccurate data collection.

### 2.3. Data Processing Procedures

The kinematics and kinetics data collected from Vicon were exported to C3D file format and then converted to coordinate system, low-pass filtered, data extraction, and formatted for kinematic and ground reaction forces (GRF) data using MATLAB (MathWorks, Massachusetts, USA). The C3D files were converted to TRC file format and mot file format using MATLAB and imported into OpenSim (Stanford University, Stanford, CA, USA) to calculate biomechanical parameters [38]. Models were scaled based on body measurements to obtain subject-specific models, and a musculoskeletal model with 23° of freedom and 92 muscle actuators was used for all musculoskeletal simulations, comparing distances between two markers on segments measured in the static standing test to distances on the generic model [39]. Subsequently, these scaling factors were applied to adjust segment length, segment inertia properties, and muscle attachment points. Measurements of muscle initiation and insertion points and muscle moment arms were aligned with the participant's limb length.

The article "The Effect of Different Degrees of Ankle Dorsiflexion Restriction on the Biomechanics of the Lower Extremity in Stop-Jumping" was published in 2024. Journal: Appl Bionics Biomech.

Static optimization algorithms were employed to estimate muscle activation and muscle force, with the results compared to surface EMG activity recorded during the experiments to validate the model. Signal-to-noise ratios were optimized through residual analysis of a subset of data from previous studies. Kinematic and kinetic data were filtered using a fourth-order zero-lag Butterworth low-pass filter with cutoff frequencies of 12 and 20 Hz, respectively. Surface EMG signals were initially band-pass filtered with a fourth-order Butterworth filter in the 10–400 Hz frequency range, followed by full-wave rectification and low-pass filtering with a cutoff frequency of 6 Hz [40]. Additionally, the EMG signals were normalized by dividing the EMG amplitude by the maximum root-mean-square (RMS) amplitude and further normalized by maximal voluntary contraction (MVC) to determine the activation level of each muscle. The muscle activation results obtained from the EMG sensors were compared with those from the musculoskeletal model simulation to assess the model's validity and accuracy. As shown in Figure 2, no significant differences were observed between muscle activation levels from the EMG data and the musculoskeletal model. Following validation, the RMS was used to quantify the degree of muscle coactivation during stop-jumping.

To compute coactivation for the descending phase of the stop-jumping, the following equation was applied [41]:

(1) $$\begin{array}{c} \text{Muscle}-\text{coactivation}\left(\%\right)=\left(\frac{\text{RMSEM}G_{antagonist}}{\text{RMSEM}G_{agonist}}\right)\times 100. \end{array}$$

The accuracy of the model was improved by using specific equations and plug-ins from the OpenSim to calculate the joint angles using the inverse kinematics algorithm, the joint torques using the inverse dynamics algorithm, and applying a residual reduction algorithm to minimize dynamic inconsistencies in the model. The inverse kinematics tool optimizes the calculation of joint angles by weighted least squares to minimize the differences between the model and experimental marker positions. Joint moments for each degree of freedom in the model were computed using the inverse kinematics tool. Joint power was then calculated as the product of angular velocity and joint moment at each time point [42]. Joint reaction analysis was used to calculate patellofemoral joint contact forces (PTF).

The PTF was estimated as a function of the knee flexion angle (x) and extensor moment (Mk) [43]. The calculation of the knee flexion angle, based on the nonlinear equation of the quadriceps arm, is outlined as follows [44]:

(2) $$\begin{array}{c} \begin{array}{c} Lq=0.00008x^{3}-0.013x^{2}+0.28x+0.046\; \end{array}. \end{array}$$

Quadriceps strength (Fq) is calculated by the following formula:

(3) $$\begin{array}{c} \begin{array}{c} Fq=\frac{Mk}{Lq}\; \end{array}. \end{array}$$

The constant *k* of the angular position (x) of the knee joint is calculated using the nonlinear equation described in [45]:

(4) $$\begin{array}{c} \begin{array}{c} K=\frac{0.462+0.00147x^{2}-0.0000384x^{2}}{\left(1-0.0162x^{2}+0.000155x^{2}-0.000000698x^{3}\right)}\; \end{array}. \end{array}$$

The PTF was computed using the quadriceps force (Fq) and a constant (k):

(5) $$\begin{array}{c} \begin{array}{c} PTF=Fq\times k\; \end{array}. \end{array}$$

The article "The Effect of Different Degrees of Ankle Dorsiflexion Restriction on the Biomechanics of the Lower Extremity in Stop-Jumping" was published in 2024. Journal: Appl Bionics Biomech.

### 2.4. Statistical Analysis

Before conducting statistical analysis, normality testing was performed on all experimental data using the Shapiro–Wilk test. If the data did not satisfy the normality criteria, the Kruskal–Wallis test was utilized to evaluate differences in kinematic and kinetic variables among different angles during the stop-jumping.

In the statistical parametric mapping (SPM) analysis, all kinematic and kinetic data from the stop-jump phase were extracted. A custom MATLAB script was used to interpolate the data points into a time series curve consisting of 101 data points, spanning from 0% to 100% of the landing [46]. Subsequently, statistical analysis was conducted using one-dimensional parameter statistical mapping program (SPM1D) scripts for one-factor repeated measures ANOVA, with a significance threshold set at 0.05. For the analysis of traditional discrete variables, MATLAB scripts were developed to extract all data from the stop-jump phase. The analyses were conducted using SPSS 27.0 for Windows software, with statistical significance determined at *p*  < 0.05 [47]. This work utilized eta-squared (*η*^2^) effect sizes to quantify the magnitude of changes in the outcome variables among different groups:

(6) $$\begin{array}{c} \begin{array}{c} \eta^{2}=\frac{{\text{SS}}_{b}}{{\text{SS}}_{t}} \end{array}. \end{array}$$

Effect size values were interpreted as follows: 0.04–0.25 indicated a small effect, 0.25–0.64 indicated a medium effect, and values greater than 0.64 indicated a large effect. Finally, the data were entered into Origin 2022 software for visualization and plotting.

## 3. Results

### 3.1. Participant Demographics

This study recruited 18 male amateur basketball and volleyball players from Ningbo University, whose mean age was 23.45 ± 1.14 years, height was 183.30 ± 4.95 cm, and weight was 80.80 ± 7.05 kg. Several inclusion criteria were employed during recruitment: (1) Participants were young and healthy amateur of basketball or volleyball at Ningbo University. (2) Young adults defined as 19–35 years old [48]. (3) Each participant engaged in basketball or volleyball activities at least three times per week, with each session lasting for a minimum of 2 hr [47]. (4) Participants had not experienced any lower limb injuries within the past 6 months and had no medical conditions that could potentially affect the experimental results [47]. (5) Participants had no history of lower limb surgery.

The article "The Effect of Different Degrees of Ankle Dorsiflexion Restriction on the Biomechanics of the Lower Extremity in Stop-Jumping" was published in 2024. Journal: Appl Bionics Biomech.

### 3.2. Results of the Kinematics and Kinetics

Figure 3 shows the difference in kinematics for the stop-jumping performed on NW, 10, and 20 W. During the stop-jumping task, as the ankle restriction angle increased, participants had an increased ankle dorsiflexion angle in the 0%–86% phase (*p*  < 0.001). In contrast, subjects had increased hip extension angles in 0%–94% phase (*p*  < 0.001); and in 66%–97% phase (*p*=0.015), the ankle restriction angle increased to 10 W; subjects had increased knee abduction angles in 11%–20% phase (*p*=0.009); and in 85%–100% phase (*p*=0.003), knee abduction angle increased; but with the increase in ankle restriction angle to 20 W, subjects had an increased knee adduction angle at and 96%–100% phase (*p*=0.016). In the 0%–100% phase, subjects had an increased knee external rotation angle (*p*  < 0.001).

During the stop-jumping task, as the angle of ankle restriction increased, subjects had increased angular velocity of ankle dorsiflexion in the 0%–27% phase (*p*  < 0.001) and ankle plantarflexion in the 34%–67% phase (*p*  < 0.001). In contrast, subjects had an increase in hip extension angular velocity at the 69%–85% phase (*p*  < 0.001), an increase in hip flexion angular velocity at the 59%–100% phase (*p*=0.001), and an increase in hip extension angular velocity only when the ankle restriction angle increased to 20 W at the 29%–36% phase (*p*=0.002). As the ankle restriction angle increased, the subject's knee flexion angular velocity increased at the 90%–100% phase (*p*=0.005); the subject's knee flexion angular velocity increased at the 0%–2% phase only when the ankle restriction angle increased to 20 W (*p*=0.015) at the 11%–15% phase; and at the 25%–38% phase and the 57%–83% phase, the knee extension angular velocity increased (*p*  < 0.001).

Table 1 shows that during the stop-jumping phase, ankle dorsiflexion angle and angular velocity (*p*  < 0.001 and *p*=0.005, respectively), ankle plantarflexion angle (*p*=0.032), knee internal and external rotation angles (*p*  < 0.001 and *p*  < 0.001, respectively), knee flexion and extension angular velocities (*p*=0.003 and *p*  < 0.001, respectively), hip extension angle and angular velocity (*p*  < 0.001 and *p*  < 0.001, respectively), and flexion angle angular velocity (*p*=0.001 and *p*  < 0.001, respectively) were significantly different between NW, 10, and 20 W.

The article "The Effect of Different Degrees of Ankle Dorsiflexion Restriction on the Biomechanics of the Lower Extremity in Stop-Jumping" was published in 2024. Journal: Appl Bionics Biomech.

Figure 4 shows the difference in kinetics for the stop-jumping performed on NW, 10, and 20 W. During the stop-jumping task, subjects had increased ankle dorsiflexion moments at the 3%–72% phase (*p*  < 0.001) as the angle of ankle restriction increased. Subjects had increased hip extension moments in the 3%–5% phase (*p*=0.016) and in the 93%–98% phase (*p*=0.005). Subjects had increased knee extension moments at the 92%–100% phase (*p*=0.005); subjects only had increased knee flexion moments at the 0%–3% phase when the ankle restriction angle was increased to 20 W (*p*=0.015); and subjects had increased knee extension moments at the 11%–14% phase, the 25%–37% phase, and the 58%–83% phase (*p*  < 0.001).

During the stop-jumping task, as the ankle restriction angle increased, subjects had increased ankle dorsiflexion power at the 7%–11% phase (*p*=0.011) and the 17%–32% (*p*  < 0.001) phase. Subjects had increased ankle plantarflexion power at the 65%–87% phase and ankle dorsiflexion power at the 93%–95% phase only when the ankle restriction angle increased to 20 W. Subjects only had increased hip flexion power at the 4%–6% phase (*p*=0.012) and at the 89%–90% phase (*p*=0.015) when the ankle restriction angle increased to 20 W. Subjects had increased knee flexion power at the 1%–7% phase (*p*=0.002) and 84%–96% phase (*p*  < 0.001), and subjects had increased knee extension power at the 12%–36% phase only when the ankle restriction angle increased to 20 W (*p*  < 0.001).

Table 2 shows that during the stop-jumping phase, ankle dorsiflexion moment and power (*p*  < 0.001 and *p*  < 0.001, respectively) plantarflexion moment and power (*p*  < 0.001 and *p*=0.024, respectively), hip extension moment (*p*=0.009), extension power and flexion power (*p*  < 0.001 and *p*  < 0.001, respectively), knee flexion moment and power (*p*  < 0.001 and *p*=0.020, respectively), and knee extension moment and power (*p*  < 0.001 and *p*  < 0.001, respectively) were significantly different between NW, 10, and 20 W.

### 3.3. Muscle Activation and Muscle Coactivation

Figure 5 shows the difference in muscle activation for the stop-jumping performed on NW, 10, and 20 W. During the stop-jumping task, subjects had increased activation of the BF at the 0%–18% phase as the ankle restriction angle increased (*p*  < 0.001); however subjects only had increased activation of the BF at the 78%–92% phase when the ankle restriction angle increased to 20 W (*p*  < 0.001). Subjects only had increased RF activation at the 22%–37% phase when the ankle restriction angle increased to 20 W (*p*  < 0.001). Subjects had increased activation of the medial and lateral femoral muscles at the 57%–71% phase (*p*  < 0.001) and decreased activation of the medial and lateral femoral muscles at the 74%–93% phase (*p*  < 0.001). There was no significant difference in the medial fibularis muscle. Activation of the lateral peroneal muscles increased at the 21%–23% phase (*p*=0.014) and decreased at the 79%–87% phase (*p*=0.001). Subjects had increased activation of the piriformis muscle at the 63%–73% phase (*p*  < 0.001) and decreased activation of the piriformis muscle at the 77%–99% phase (*p*  < 0.001). Activation of the TA muscle increased in the 84%–96% phase (*p*  < 0.001).

The article "The Effect of Different Degrees of Ankle Dorsiflexion Restriction on the Biomechanics of the Lower Extremity in Stop-Jumping" was published in 2024. Journal: Appl Bionics Biomech.

Figure 6 shows the difference in muscle coactivation for the stop-jumping performed on NW, 10, and 20 W. As the limiting angle of ankle mobility increases, SOL/TA and MG/TA gradually decrease and BF/RF and BF/VM gradually increase.

### 3.4. Muscle Force

Figure 7 shows the difference in muscle force for the stop-jumping performed with NW, 10, and 20 W. During the stop-jumping task, as the angle of ankle restriction increased, subjects showed an increase in muscle strength of the BF at the 0%–17% phase (*p*  < 0.001) and a decrease in muscle strength of the BF at the 78%–91% phase (*p*  < 0.001). However, at the 68%–70% phase, only the BF activation increased when the angle of ankle restriction was increased to 20 W (*p*=0.017). Subjects had increased muscle strength of the RF at the 26%–34% phase (*p*=0.001); however at the 52%–56% phase, only the RF muscle strength decreased when the ankle restriction angle increased to 10 W (*p*=0.004), and at the 6%–15% phase, only the RF muscle strength decreased when the ankle restriction angle increased to 20 W (*p*  < 0.001). The muscle strength of the medial femoral muscle decreased during the 76%–90% phase (*p*  < 0.001) and increased in the 97.5%–100% phase only when the ankle restriction angle increased to 20 W (*p*  < 0.001). Muscle strength of the lateral femoral muscles increased during the 64%–68% phase (*p*=0.005), decreased during the 75%–91% phase (*p*  < 0.001), and increased during the 94%–100% phase only when the ankle restriction angle increased to 20 W (*p*=0.002). Subjects only had a decrease in muscle strength of the MG at the 83%–85.5% phase when the ankle restriction angle increased to 20 W (*p*=0.011) and an increase in muscle strength of the MG at the 83%–85.5% phase (*p*  < 0.001). Subjects only had an increase in ankle restriction angle to 20 W at the 16%–22% phase (*p*=0.002) and the 91%–98% phase (*p*  < 0.001) with an increase in lateral gastrocnemius muscle strength (*p*=0.011) and a decrease in lateral gastrocnemius muscle strength at the 83%–86% phase (*p*  < 0.001). Muscle strength of the SOL decreased in the 34%–38% (*p*=0.004) and 77%–89% (*p*  < 0.001) phases, increased in the 63%–68% phase only when the ankle restriction angle increased to 10 W (*p*=0.006), and increased in the 91%–100% phase only when the ankle restriction angle increased to 20 W (*p*  < 0.006) and muscle strength increased (*p*  < 0.001). Muscle strength of the TA muscle increased in the 83.5%–96.7% phase (*p*  < 0.001).

The article "The Effect of Different Degrees of Ankle Dorsiflexion Restriction on the Biomechanics of the Lower Extremity in Stop-Jumping" was published in 2024. Journal: Appl Bionics Biomech.

Table 3 shows that during the stop-jumping phase, BF muscle force (*p*  < 0.001), RF muscle force (*p*  < 0.001), VM muscle force (*p*=0.005), vastus lateralis muscle force (*p*  < 0.001), SOL muscle force (*p*=0.017), and TA muscle force (*p*=0.003) were significantly different between NW, 10, and 20 W.

### 3.5. Patellofemoral Joint Contact Force

Figure 8 shows the difference in PTF for stop-jumping performed with NW, 10, and 20 W. During the stop-jumping task, PTF increased progressively as the angle of ankle restriction increased in subjects at the 3%–8% phase (*p*=0.015).

## 4. Discussion

This study revealed that modifying ankle joint mobility can lead to adaptive changes in the knee joint. Prior research has demonstrated that restrictions in ankle mobility correlate with alterations in knee sagittal and frontal plane kinematics [20]. As the limitations of ankle dorsiflexion mobility change, athletes may adjust their movement strategies, such as through greater hip and knee mobility to compensate for the limitations during movements like stop-jumping.

In terms of kinematic outcomes, previous studies have shown that ankle valgus angles and angular velocities typically increase during stopped jumps in amateur male basketball players [17] and lower peak ankle dosiflexion angles are associated with patellar tendinopathy [23]. Our findings revealed that with increasing restriction angles at the ankle joint, participants displayed greater ankle dorsiflexion angles and higher dorsiflexion angular velocities during stop-jumping. Previous studies have demonstrated that ankle dorsiflexion excursion is negatively correlated with the peak vertical ground reaction force loading rate and positively correlated with the peak ankle flexor plantar moment [49], potentially in response to increased loading during the jumping maneuver. These heightened ankle dorsiflexion metrics may aid in better absorption of impact forces and improved jump propulsion, accompanied by compensatory adjustments during the jump phase such as increased knee and hip extension angles and angular velocities. These compensatory adaptations could help athletes overcome the limitations imposed by restricted ankle joint motion and enhance jumping efficiency. Previous studies investigating muscle activity in response to external moments during single-leg landings in adolescent basketball players have found that internal rotation of the knee is associated with an increased risk of knee injury [50], and in a video analysis of injury footage examining the mechanisms of noncontact ACL injuries, it was found that inward tibial rotation after a landing resulted in an ACL tear [51]. A reduction in knee internal rotation contributes to improved core control, which may reduce the risk of ACL injury [52]. Our findings suggest that knee internal rotation is observed when jumping on a flat surface, which may lead to decreased knee stability and thus knee injury, but normalizes as the ankle restriction angle increases, suggesting that the body's strategy involves adjusting the other joint angles according to the ankle restriction to maintain stability. Therefore, we recommend that individuals with poor knee stability or knee injuries consider jump training on a moderate wedge board to help optimize joint mechanics and reduce the risk of injury.

The article "The Effect of Different Degrees of Ankle Dorsiflexion Restriction on the Biomechanics of the Lower Extremity in Stop-Jumping" was published in 2024. Journal: Appl Bionics Biomech.

In terms of kinetic outcomes, prior studies have shown that increased strength derived from high-speed knee and hip extension contributes to enhanced vertical jump performance [53, 54, 55]. This conclusion was reached by testing the force–velocity characteristics of knee–hip extension and vertical jumps in 67 untrained subjects and nine males, under conditions of fast jumps and further unilateral isometric knee initial angle jumps. Our study found that as the angle of ankle restriction increased, participants exhibited higher hip and knee extension moments and forces. This adaptation may represent a compensatory mechanism in response to the limitations imposed by ankle restrictions on ROM and force transmission. By augmenting hip and knee extension torque and strength, participants were able to execute jumping maneuvers more effectively despite ankle restrictions. A prior study employing an adaptive neurofuzzy inference system to estimate ankle angles in a healthy population has established that kinematic variations of the ankle joint in the sagittal, coronal, and horizontal planes may be associated with the development of knee osteoarthritis [56, 57]. Furthermore, our study observed that as the angle of ankle restriction increased, participants demonstrated increased flexion and extension torque and force at the knee. This heightened lower extremity muscle activity likely reflects a strategy to offset the impact of ankle joint restriction during jumping maneuvers.

The article "The Effect of Different Degrees of Ankle Dorsiflexion Restriction on the Biomechanics of the Lower Extremity in Stop-Jumping" was published in 2024. Journal: Appl Bionics Biomech.

The knee joint is crucial for maintaining body balance [14, 58], and PTF is a critical factor in knee stability [59]. The patella functions as a mechanical pulley, enhancing the lever arm of the quadriceps tendon and thereby increasing the efficiency of the quadriceps muscle during knee extension [43]. Moreover, the patella serves to prevent lateral and medial patellar dislocation and offers stability during knee flexion and extension movements. Increasing the contact force between the patella and femur contributes significantly to knee joint stabilization. This contact force occurs within the knee joint structure between the femur and tibia. Augmenting the contact force between the patella and femur leads to a broader contact area or more uniform force distribution, thereby reducing stress on specific areas and enhancing overall knee joint stability. Through prior research, we were able to calculate the PTF for study participants [44, 45, 60]. Prior studies have established that an increase in PTF relative to joint surface area signifies a larger contact area or a more uniform distribution of force [61, 62, 63], potentially reducing site-specific stresses and enhancing knee stability. Our results revealed a gradual increase in PTF in subjects as the ankle joint restriction angle increased. This finding suggests that the biomechanical characteristics of the lower extremity adapt in response to changes in ankle joint restriction angles, which could positively impact the patellofemoral joint.

Joint stability is not only influenced by contact forces between knee bones but also significantly affected by muscle coactivation. Impaired muscle coactivation can result in reduced knee stability. The pattern of muscle coactivation surrounding the knee joint plays a vital role in providing dynamic knee stability and preventing injuries [64]. Muscle coactivation helps to convert valgus forces into joint contact forces, thereby safeguarding the knee from injury [65]. Expanding on previous research, our study analyzed and quantified the muscle coactivation patterns around the knee joints of our participants [41]. Research has emphasized that the stability of lower limb joints heavily depends on the coordinated coactivation of muscles [41, 64, 66, 67, 68]. Ankle joint mobility limitation results in decreased SOL and MG muscle activation, alongside increased activation of the TA muscle. Our findings revealed that as ankle mobility restriction increased, the ratios of SOL/TA and MG/TA progressively decreased, while the ratios of BF/RF and BF/VM progressively increased. These changes suggest that heightened ankle restriction may enhance knee stability and muscle control. This aligns with prior research indicating that coordinated knee muscle activation supports joint stiffness and shields the ACL from injury by transforming valgus forces into joint contact forces [68]. Adaptive responses were noted under various bracing conditions during stop-jumping on 10 and 20 W, potentially influencing subjects' stability maintenance. While knee angles did not significantly change, adaptations in muscle coactivation were observed, which significantly contributed to stability maintenance under limited ankle mobility conditions. Previous studies have emphasized the close link between changes in muscle strength and changes in kinematic and kinetic characteristics [69, 70, 71, 72]. Our results found significant adjustments in peak strength of several muscles as the angle of ankle restriction increased. These changes may reflect adaptive and compensatory strategies of muscle strength aimed at adapting to ankle restriction conditions to maintain stability and movement efficiency. Specifically, peak muscle strength of the BF, RF, lateral femoris, medial femoris, SOL, and TA appeared to change significantly at different stages as the angle of ankle restriction increased.

The article "The Effect of Different Degrees of Ankle Dorsiflexion Restriction on the Biomechanics of the Lower Extremity in Stop-Jumping" was published in 2024. Journal: Appl Bionics Biomech.

These results confirm our initial hypothesis and provide valuable insights into how ankle restrictions affect biomechanical adaptations during jump stopping. They deepen our understanding of how different degrees of ankle restriction impact athletic performance from a biomechanical perspective. Overall, this study enhances our comprehension of the biomechanical effects of ankle joint restriction during sharp stop-jump maneuvers. By elucidating the lower extremity's adaptive response to ankle joint restriction, these findings may inform targeted interventions aimed at optimizing athletic efficiency and reducing injury risk among athletes. However, there are some limitations to the current study, which is the lack of research on limiting ankle dorsiflexion mobility during a sharp stop and jump by gender, as well as the current study that investigated the effect of limiting ankle dorsiflexion mobility during a sharp stop and jump; therefore further research is planned in the future to include female participants and will take a different movement scenario limiting ankle dorsiflexion mobility to validate and extend the current findings.

## 5. Conclusions

In conclusion, our study analyzes and compares stopping jumps performed with varying degrees of ankle restriction by quantifying the kinetic and kinematic changes during the stopping phase. From the results, it was observed that as the degree of ankle dorsiflexion angle restriction increased, the coactivation of the muscles around the knee joint increased and the PTF increased, probably because when the ankle dorsiflexion angle is restricted, one cannot adequately adjust one's body to adapt to the balance. Whereas the knee joint is a key part of the body that plays an important role in maintaining balance, the increased degree of muscle coactivation around the knee joint and the increased PTF may be a compensatory response to the body's adaptive adjustment to balance. Further studies should focus on the biomechanical effects of limiting ankle mobility on different maneuvers to validate our findings.

The article "The Effect of Different Degrees of Ankle Dorsiflexion Restriction on the Biomechanics of the Lower Extremity in Stop-Jumping" was published in 2024. Journal: Appl Bionics Biomech.

## Figures and Tables

**Figure 1:** (a) Illustration of the schematic representation of reflective marker placement on body skeletal landmarks. (b) Illustration of the position of an EMG test on a human lower limb. (c) Illustration of the stop-jumping biomechanical test process.

**Figure 2:** Illustration of EMG muscle activation, the red line represents the EMG muscle activation results, and the blue shaded area represents the muscle activation results in the musculoskeletal model. The vertical scale ranges from 0 to 1, indicating muscle activation levels from none to full. The horizontal scale ranges from 0 to 100, representing the stance phase.

**Figure 3:** Means to the kinematics of the ankle, knee, and hip joints during the stop-jumping. The results of the SPM for NW, 10, and 20 W are shown in the figure. The blue, red, and purple lines represent the results of the SPM analyses for NW and 10 W, 10 W and 20 W, and NW and 20 W, respectively. *F* ^*∗*^ is a specific threshold to distinguish between the region of significance and the region of non-significance.

**Figure 4:** Means to the kinetics of the ankle, knee, and hip joints during the stop-jumping. The results of the SPM for NW, 10, and 20 W are shown in the figure. The blue, red, and purple lines represent the results of the SPM analyses for NW and 10 W, 10 W and 20 W, and NW and 20 W, respectively. *F* ^*∗*^ is a specific threshold to distinguish between the region of significance and the region of non-significance.

**Figure 5:** Mean ± SD normalized time-series muscle activation during the stop-jumping. The results of the SPM for NW, 10, and 20W are shown in the figure. The blue, red, and purple lines represent the results of the SPM analyses for NW and 10W, 10W and 20W, NW and 20W, respectively, “ ^*∗*^” indicates the critical value to determine whether the statistical results are statistically significant or not, when the *F*-value exceeds this critical value, it means that there is a statistically significant difference in that region.

The article "The Effect of Different Degrees of Ankle Dorsiflexion Restriction on the Biomechanics of the Lower Extremity in Stop-Jumping" was published in 2024. Journal: Appl Bionics Biomech.

**Figure 6:** Illustration of lower limb muscle coactivation results for NW, 10, and 20 W during the stop-jumping. *Abbreviations*. TA, tibialis anterior; MG, medial gastrocnemius; BF, biceps femoris; RF, rectus femoris; VM, vastus medialis; SOL, soleus.

**Figure 7:** Mean ± SD normalized time-series muscle force during the stop-jumping. The results of the SPM for NW, 10, and 20W are shown in the figure. The blue, red, and purple lines represent the results of the SPM analyses for NW and 10W, 10W and 20W, NW and 20W, respectively, “ ^*∗*^” indicates the critical value to determine whether the statistical results are statistically significant or not, when the *F*-value exceeds this critical value, it means that there is a statistically significant difference in that region.

**Figure 8:** Mean ± SD normalized time series of patellofemoral joint contact forces during the stop-jumping. The results of the SPM for NW, 10, and 20 W are shown in the figure. The blue, red, and purple lines represent the results of the SPM analyses for NW and 10 W, 10 W and 20 W, and NW and 20 W, respectively. *F* ^*∗*^ is a specific threshold to distinguish between the region of significance and the region of non-significance.

**Table 1:** Detailed results of peak joint angles and velocities of subjects performing stop-jumping at NW, 10, and 20 W.

Parameters	Peak value	NW (mean ± SD)	10 W (mean ± SD)	20 W (mean ± SD)	*p*-value	*F*	*ES*
Ankle angle (°)	Dorsiflexion	23.70 ± 4.27	28.01 ± 3.66	31.76 ± 2.32	＜0.001 ^*∗*^	183.928	0.820
	Plantarflexion	−31.64 ± 8.30	−27.78 ± 9.81	−27.66 ± 11.97	0.032 ^*∗*^	3.578	0.081

Ankle velocity (°/s)	Dorsiflexion	−145.14 ± 24.39	−147.35 ± 27.50	−148.68 ± 34.46	0.710	0.343	0.004
	Plantarflexion	955.58 ± 134.10	910.07 ± 194.68	991.85 ± 138.32	0.005 ^*∗*^	5.546	0.112

Hip angle (°)	Flexion	61.89 ± 7.53	62.26 ± 8.40	60.70 ± 8.06	0.001 ^*∗*^	6.859	0.071
	Extension	6.80 ± 5.28	9.32 ± 4.34	7.25 ± 4.60	＜0.001 ^*∗*^	15.141	0.254

Hip velocity (°/s)	Flexion	−195.76 ± 58.16	−229.10 ± 53.70	−162.84 ± 46.08	＜0.001 ^*∗*^	74.469	0.594
	Extension	427.35 ± 72.88	373.77 ± 73.34	340.75 ± 45.64	＜0.001 ^*∗*^	58.143	0.533

Knee angle (°)	Flexion	−85.46 ± 7.46	−83.83 ± 11.23	−85.63 ± 11.65	0.276	1.307	0.028
	Extension	−11.29 ± 6.23	−11.98 ± 8.78	−10.98 ± 9.21	0.688	0.374	0.004
	Adduction	−1.07 ± 1.33	−1.40 ± 2.01	−1.07 ± 1.80	0.328	1.127	0.022
	Abduction	5.58 ± 2.79	5.63 ± 2.06	5.65 ± 2.34	0.986	0.014	0.001
	Internal rotation	5.36 ± 0.91	4.46 ± 1.12	2.39 ± 1.22	＜0.001 ^*∗*^	42.575	0.834
	External rotation	−3.18 ± 1.05	−4.04 ± 1.23	−5.80 ± 1.42	＜0.001 ^*∗*^	19.713	0.523

Knee velocity (°/s)	Flexion	424.38 ± 80.07	436.59 ± 75.00	401.93 ± 88.33	0.003 ^*∗*^	5.906	0.059
	Extension	−966.17 ± 92.94	−898.33 ± 109.14	−874.30 ± 79.56	＜0.001 ^*∗*^	84.835	0.643

*Note*. “ ^*∗*^” indicates a significant difference (*p*  < 0.05) between NW, 10, and 20 W for the stop-jumping phase.

The article "The Effect of Different Degrees of Ankle Dorsiflexion Restriction on the Biomechanics of the Lower Extremity in Stop-Jumping" was published in 2024. Journal: Appl Bionics Biomech.

**Table 2:** Detailed results of joint moments and power for subjects performing stop-jumping at NW, 10, and 20 W.

Parameters	Peak value	NW (mean ± SD)	10 W (mean ± SD)	20 W (mean ± SD)	*p*-value	*F*	*ES*
Ankle moment (Nm/kg)	Dorsiflexion	0.25 ± 0.05	0.16 ± 0.05	0.08 ± 0.06	＜0.001 ^*∗*^	68.690	0.725
	Plantarflexion	−1.98 ± 0.23	−2.11 ± 0.32	−2.18 ± 0.22	＜0.001 ^*∗*^	9.193	0.261

Ankle power (W/kg)	Dorsiflexion	13.33 ± 1.53	13.63 ± 1.13	15.36 ± 1.30	＜0.001 ^*∗*^	26.429	0.504
	Plantarflexion	−2.37 ± 1.02	−2.90 ± 0.86	−2.77 ± 0.84	0.024 ^*∗*^	4.024	0.134

Hip moment (Nm/kg)	Flexion	0.91 ± 0.51	0.85 ± 0.54	1.02 ± 0.73	0.320	1.163	0.039
	Extension	−2.67 ± 1.18	−2.59 ± 1.02	−2.99 ± 1.32	0.009 ^*∗*^	5.113	0.150

Hip power (W/kg)	Flexion	5.40 ± 2.13	5.49 ± 2.06	6.26 ± 2.39	＜0.001 ^*∗*^	8.622	0.242
	Extension	−9.77 ± 5.71	−7.73 ± 4.73	−5.18 ± 3.54	＜0.001 ^*∗*^	16.831	0.384

Knee moment (Nm/kg)	Flexion	−0.54 ± 0.31	−0.30 ± 0.25	−0.29 ± 0.23	＜0.001 ^*∗*^	12.547	0.309
	Extension	2.85 ± 0.30	2.76 ± 0.40	2.52 ± 0.46	＜0.001 ^*∗*^	11.974	0.300

Knee power (W/kg)	Flexion	15.95 ± 2.07	16.05 ± 2.33	14.46 ± 2.63	0.020 ^*∗*^	4.652	0.288
	Extension	−11.64 ± 2.83	−9.88 ± 1.89	−9.52 ± 3.45	＜0.001 ^*∗*^	12.037	0.511

*Note*. “ ^*∗*^” indicates a significant difference (*p*  < 0.05) between NW, 10, and 20 W for the stop-jumping phase.

**Table 3:** Detailed results of muscle force for subjects performing stop-jumping at NW, 10, and 20 W.

Muscle force parameters (BW)	NW (Mmean ± SD)	10W (mean ± SD)	20 W (mean ± SD)	*p*-value	*F*	*ES*
Biceps femoris	1.83 ± 0.34	2.52 ± 0.18	2.91 ± 0.42	＜0.001 ^*∗*^	18.272	0.723
Rectus femoris	11.75 ± 1.64	13.62 ± 2.17	14.17 ± 1.90	＜0.001 ^*∗*^	14.468	0.559
Vastus medialis	1.60 ± 0.20	1.91 ± 0.24	1.82 ± 0.13	0.005 ^*∗*^	6.844	0.406
Vastus lateralis	2.57 ± 0.34	3.31 ± 0.25	3.06 ± 0.30	＜0.001 ^*∗*^	18.778	0.591
Medial gastrocnemius	1.51 ± 0.12	1.47 ± 0.18	1.40 ± 0.16	0.246	1.505	0.131
Lateral gastrocnemius	0.77 ± 0.11	0.77 ± 0.16	0.72 ± 0.09	0.523	0.666	0.053
Soleus	1.73 ± 0.25	2.16 ± 0.32	1.84 ± 0.21	0.017 ^*∗*^	5.301	0.399
Tibialis anterior	1.97 ± 0.24	2.34 ± 0.42	2.38 ± 0.20	0.003 ^*∗*^	7.673	0.434

*Note*. “ ^*∗*^” indicates a significant difference (*p*  < 0.05) between NW, 10, and 20 W for the stop-jumping phase.

## Data Availability

All data relevant to the current study are included in the article; further inquiries can be directed to the corresponding author.
